RETRACTED

# Effect of Shugan Jianpi Recipe Combined with Cross Moxibustion on Biochemical Examination Indexes and Total Score of TCM Symptoms in Patients with Spleen-Stomach Damp-Heat Diarrhea Irritable Bowel Syndrome

**DOI:** 10.1155/2022/8286146

**Published:** 2022-04-23

**Authors:** Di Liu, Meiying Ruan, Chenghui Tong, Rongrong Huang

**Affiliations:** ^1^Shengzhou People's Hospital (Shengzhou Branch of the First Hospital of Zhejiang University) Department of Traditional Chinese Medicine, 312400, China; ^2^Shengzhou City Changle Town Central Health Center Acupuncture Department, Shengzhou City 312467, China; ^3^Yuyao Hospital of Traditional Chinese Medicine, Yuyao City 315400, China; ^4^Shengzhou People's Hospital (Shengzhou Branch of the First Hospital of Zhejiang University) Urology Department, 312400, China

## Abstract

**Objective:**

To explore the effect of Shugan Jianpi recipe combined with cross moxibustion on biochemical examination indexes and total score of TCM symptoms in patients with spleen-stomach damp-heat diarrhea irritable bowel syndrome (IBS).

**Methods:**

Sixty patients with spleen-stomach damp-heat diarrhea (IBS) treated in our hospital from January 2019 to September 2021 were enrolled. The patients were randomly assigned into the control group and study group. The control group was treated with Chang Shugan Jianpi recipe, and the study group was treated with Shugan Jianpi recipe combined with cross moxibustion. The curative effect, single symptom score, total score of TCM clinical symptoms, plasma gastrointestinal hormone level, IBS-QOL score, and recurrence were compared.

**Results:**

First of all, we compared the curative effects. The study group was significantly effective in 24 cases, effective in 5 cases, and ineffective in 1 case, and the effective rate was 96.67%. In the control group, 13 cases were markedly effective, 10 cases were effective, and 7 cases were ineffective, and the effective rate was 76.67%. The effective rate of the study group was higher compared to the control group (*P* < 0.05). Secondly, the individual symptom scores were compared. Compared between the two groups, the scores of diarrhea times, stool characteristics, abdominal pain, and abdominal distension in the study group were lower compared to the control group (*P* < 0.05). After treatment, the total score of TCM clinical symptoms decreased. Compared between the two groups, the total score of TCM clinical symptoms in the study group was lower compared to the control group at 1 week, 2 weeks, and 4 weeks after treatment (*P* < 0.05). After treatment, the levels of 5-HT and VIP decreased. The levels of 5-HT and VIP in the study group were lower compared to the control group (*P* < 0.05). The scores of anxieties, health worry, behavioral disorder, social reaction, somatic intention, interpersonal relationship, dietary concern, and sexual behavior in the study group were lower compared to the control group. The IBS-QOL scores were significantly lower compared to the control group (*P* < 0.05). Finally, we compared the recurrence. The recurrence rate in the study group was lower compared to the control group (*P* < 0.05).

RETRACTED

**Conclusion:**

The prescription combined with cross moxibustion has the effect of soothing the liver and invigorating the spleen, resolving dampness and stomach, and can reduce the main clinical symptoms of patients with diarrhea IBS of spleen-stomach damp-heat type, and the overall effect is significant. It can also enhance the emotional state of anxiety and depression and achieve the overall psychological and physical balance and health state, and the recurrence rate is low, which can be further applied in clinic.

## 1. Introduction

Irritable bowel syndrome (IBS) is a common functional gastrointestinal disease characterized by abdominal pain and discomfort and changes in intestinal function [1]. According to Rome IV, the diagnostic criteria of IBS are defined as follows: (1) Recurrent abdominal pain occurred at least 6 months before the diagnosis of IBS, and abdominal pain occurred at least one day a week for the last 3 months, accompanied by two or more of the following abnormal changes: (1) related to defecation, (2) accompanied by changes in defecation frequency, and (3) accompanied by changes in fecal traits (appearance). (2) Other intestinal organic lesions such as Crohn's disease, ulcerative colitis, and intestinal tumors were excluded by colonoscopy or pathological examination. According to the difference of stool characters, IBS can be assigned into constipation type (IBS-C), diarrhea type (IBS-D), mixed type (IBS-M), and uncertain type (IBS-U). In recent years, the research in China has increased year by year [2, 3]. Current studies have indicated that the occurrence of IBS-D is related to visceral sensitivity, gastrointestinal motility disorders, gastrointestinal hormones and neuropeptides or brain-intestinal aspiration mechanism, flora disorders, and intestinal infection, as well as psychosocial factors (such as anxiety and depression), sleep disorders, and irregular diet [4]. Traditional Chinese medicine (TCM) does not have the name of “IBS.” According to its clinical symptoms, modern Chinese medicine mostly classifies it as “diarrhea” or “abdominal pain,” sometimes also called “diarrhea” [5]. There is stomach discharge, spleen discharge, large intestine discharge, small intestine discharge, and big diarrhea, which is called Hou Zhong [4, 5]. This nomenclature continued to the Sui and Tang dynasties, and the reference to blood dysentery in “various causes and symptoms of dysentery” pointed out: “Blood permeates into the intestine, intestinal deficiency leads to diarrhea, so it is also blood dysentery”, that is, diarrhea, which gives rise to the name of “dysentery.”

RETRACTED

At present, there is no unified regulation on the dialectical classification of diarrhea IBS. In the consensus of TCM experts on diagnosis and treatment of IBS published in 2017, IBS-D is assigned into liver depression and spleen deficiency, spleen deficiency and dampness, spleen and stomach damp-heat, spleen and kidney yang deficiency, and cold and heat mixed syndrome [6]. According to the guidelines for diagnosis and treatment of Digestive Diseases of TCM in 2006, the disease is assigned into spleen and stomach deficiency type, liver depression and spleen deficiency type, liver depression and qi stagnation type, spleen and stomach damp-heat type, and spleen and kidney yang deficiency type [7]. In IBS-D spleen deficiency and dampness syndrome of TCM treatment, not only internal medicine effect is very good; external treatment is also a great advantage. It is pointed out that the external treatment method makes the drug act directly on the skin and mucosa, through local absorption, so as to achieve the purpose of treatment; the commonly used external treatment methods are acupuncture, acupoint application, moxibustion, TCM enema, and acupoint injection [7, 8]. Moxibustion can stimulate the function of meridians and collaterals by stimulating corresponding acupoints and sites and then adjust the state of the body to achieve the purpose of disease treatment and prevention. “Lingshu function” has long been the view that “what acupuncture does not do, it is appropriate to moxibustion” [6, 9]. Cross moxibustion produces warm stimulation to the body by burning moxa velvet, which plays the role in warming meridians, dispelling cold and relieving pain, tonifying qi, activating blood circulation, dispelling cold, and dehumidification. Coupled with the role of moxa leaves themselves, moxa leaves are bitter, pungent, and warm, with the functions of warming menstruation and dispelling cold, relieving pain, and hemostasis [9]. Liang Tao Hongjing's “Records of famous doctors” makes a comprehensive discussion on its medicinal theory: “moxa leaves, moxibustion all kinds of diseases” [10]. However, there are few reports on the treatment of spleen-damp-heat diarrhea IBS with Shugan Jianpi recipe combined with cross moxibustion in the past. Based on this, our study discussed the clinical effect of Shugan Jianpi recipe combined with cross moxibustion in the treatment of spleen-stomach damp-heat diarrhea IBS.

RETRACTED

## 2. Patients and Methods

### 2.1. General Information

Sixty patients with spleen-stomach damp-heat diarrhea IBS treated in our hospital from January 2019 to September 2021 were enrolled. The patients were randomly assigned into the control group and study group. The control group was treated with Chang Shugan Jianpi recipe, and the study group was treated with Shugan Jianpi recipe combined with cross moxibustion. In the control group, the age was 25-74 years, with an average age of 45.75 ± 3.44 years, including 17 males and 13 females, while in the study group, the age was 24-76 years with an average age of 45.96 ± 3.78 years, including 16 males and 14 females. There exhibited no statistical significance in the general data. This study was permitted by the Medical Ethics Association of our hospital, and all patients signed informed consent.

#### 2.1.1. Diagnostic Criteria

Western diagnostic criteria: (1) IBS Rome IV diagnostic criteria 12 indicated recurrent abdominal pain with an average of at least 1 day a week in the past three months, accompanied by at least two of the following three items: (1) related to defecation, (2) accompanied by changes in defecation frequency, and (3) accompanied by changes in fecal characteristics (appearance). Note: before being enrolled in this study, patients developed symptoms for 6 months and nearly 3 months met the above criteria. (2) Rome IV diagnostic criteria of diarrhea IBS (IBS-D): in addition to the above diagnostic criteria, it should also meet the “>25% stool trait type 6 or 7 bristol stool character type 6 or 7, and <25% stool type 1 or 2 type” can be diagnosed

Diagnostic criteria of TCM: refer to the consensus on TCM diagnosis and treatment of IBS (2017) [11] and “consensus of TCM experts on diagnosis and treatment of diarrhea” (2017) [12]. Diagnostic criteria of spleen deficiency and dampness syndrome: main symptoms: (1) diarrhea, (2) faint abdominal pain, and (3) diarrhea in stool and secondary symptoms: (1) fear of food and cold, (2) fatigue and drowsiness; and (3) stupefied; tongue and pulse: light tongue, tooth marks on the edge, white and greasy fur; pulse weakness; syndrome diagnosis requirements: two main symptoms, two additional symptoms, reference to tongue and pulse, can be diagnosed

Inclusion criteria: (1) patients who meet the diagnostic criteria of IBS-D Rome IV in western medicine; (2) patients who meet the syndrome diagnostic criteria of spleen deficiency and dampness syndrome in TCM; (3) patients' age ranged from 18 to 65 years; (4) patients did not take antidiarrheal drugs or antibiotics or other related drugs that affect the clinical study within 30 days; (5) voluntarily participate in this clinical study and agree to accept relevant treatment and examination and can adhere to the follow-up; and (6) voluntarily sign the informed consent form for this test

Exclusion criteria: (1) those who did not meet the above inclusion criteria; (2) pregnant women, lactating women, and those who prepared for pregnancy; (3) organic lesions such as intestinal mucosal erosion, bleeding, and intestinal tumors confirmed by colonoscopy or pathology; (4) those complicated with severe primary diseases such as cardiocerebrovascular system, hematopoietic system, and endocrine system and need to take medication for a long time; (5) allergic physique; and (6) those who were unable to express subjective discomfort

Termination criteria: (1) patients with serious side effects during treatment or other diseases that affect the observation of the trial should be terminated according to the doctor's judgment; (2) there was a serious deviation in the implementation of the clinical trial program (for example, the compliance was too poor to evaluate the drug effect); and (3) those who were unable to continue and voluntarily withdraw from the clinical trial due to personal reasons

RETRACTED

### 2.2. Treatment Methods

Control group: Codonopsis pilosula 15 g, Atractylodes macrocephala 10 g, Poria 15 g, Bupleurum 10 g, Radix Paeoniae Alba 15 g, Radix Astragali 20 g, Pinellia ternata 10 g, tangerine peel 6 g, Salvia miltiorrhiza 10 g, fried lentil 15 g, Fructus Aurantii 10 g, licorice 10 g. And with the disease: diarrhea symptoms seriously affect the quality of life of patients can add Euryale 15 g, nutmeg 15 g; those who cannot sleep at night change Poria into Poria; those with poor stomach fire add 6 g of Coptis chinensis, 3 g of Evodia rutaecarpa; those with obvious liver depression and qi stagnation add 15 g and increase the dosage of Bupleurum and tangerine peel, etc. Usage: use the TCM room machine in our hospital with nondecoction granule preparation (Jiangyin Tianjiang Pharmaceutical Co., Ltd.) and take it separately after breakfast and dinner every day.

The study group was treated with Shugan Jianpi recipe combined with cross moxibustion, and the Shugan Jianpi recipe was the same as the control group. Cross moxibustion: (1) selection of acupoints: take Shenque acupoint as the center, open 4 inches to the upper and lower left and right sides, that is, up to Zhongwan, down to Zhongji, and left and right to Dazheng; (2) disinfection: disinfect with 75% alcohol cotton balls; (3) mulberry paper: covered with mashed ginger, wide 3 cm, high 2.5 cm, narrow at the top and wide at the bottom; (4) place the moxa, and the moxa is measured by the inch of the same body; (5) ignition: the sequence starts from Shenque and then ignites up, down, left, and right; (6) replace the second strong after one strong moxibustion, 2 strong for each moxibustion, and 3 strong for severe moxibustion; and (7) after moxibustion, remove the mashed ginger and moxa ash and clean the moxibustion area. Moxa ash and ginger foam were wiped off with hot towels once a week for 4 weeks. Telephone follow-up visits were made to ensure patient compliance.

RETRACTED

Both two groups were treated continuously for 4 weeks, and the changes of the subjects' condition before and after treatment were observed, respectively. During the study, other drugs that had effects on the stomach and intestines were discontinued. During the treatment, patients in both groups should abstain from drinking, adhere to a regular diet, avoid eating cold, spicy, and irritating food, and try to keep a good mood; the two groups are at the end of the course of treatment result statistics, so as to evaluate the curative effect.

### 2.3. Observation Index

#### 2.3.1. IBS-SSS Evaluation Standard of Curative Effect

(1) Significant effect: after the end of the course of treatment, the symptom grade was reduced by 2 grades. (2) Effective: after the end of the course of treatment, the symptom grade was reduced by 1 grade. (3) Invalid: those who fail to meet the above standards. Refer to the guiding principles of Clinical Research on New drugs of TCM.

#### 2.3.2. Evaluation of the Curative Effect of Single Symptom

Refer to the guiding principles of Clinical Research on New drugs of TCM in 2002 [13]. (1) Clinical recovery: after the end of the course of treatment, the symptoms disappeared. (2) Significant effect: after the end of the course of treatment, the symptom grade was reduced by 2 grades. (3) Effective: after the end of the course of treatment, the symptom grade was reduced by 1 grade. (4) Invalid: those who fail to meet the above standards. Note: the symptom classification refers to the quantitative standard of symptom classification in Table 1.

#### 2.3.3. Criteria for Judging the Curative Effect of TCM Symptoms

The evaluation standard of TCM symptom score is based on the scoring rules formulated by the guiding principles for Clinical Research of New drugs of TCM (trial) issued by the Administration of TCM in 2002 and the consensus of TCM experts in diagnosis and treatment of IBS [14]. The score was according to the severity of the disease. The main symptoms such as diarrhea, abdominal pain, and stool rot were counted according to normal, mild, moderate, and severe points (0, 2, 4, and 6 points, respectively); fear of eating, fatigue, and drowsiness were counted as secondary symptoms according to normal, mild, moderate, and severe symptoms (0 points, 1 point, 2 points, and 3 points). For tongue and pulse as a reference, the higher the score, the more serious the symptoms, and the main symptom score and secondary score were added as the total symptom score.

RETRACTED

#### 2.3.4. Detection of Plasma Gastrointestinal Hormones

Before and after treatment, the patients' fasting elbow venous blood 5 mL was collected and placed for 1 hour. The supernatant was centrifuged with 3000 r/min 10 min (centrifugal radius 10 cm) at 4°C, and the supernatant was put into the refrigerator at -20°C for detection. The expression levels of 5-hydroxytryptamine (5-HT) and vasoactive intestinal peptide (VIP) were detected by enzyme-linked immunosorbent assay (ELISA). The procedure of the kit was strictly followed by special personnel.

#### 2.3.5. IBS-QOL Scoring

A total of 34 items were recorded from 8 dimensions: anxiety, health worry, behavioral disorder, social response, physical intention, interpersonal relationship, dietary concern, and sexual behavior [15]. The severity was divided into normal, mild, moderate, and severe scores of 1-5. The higher the score, the worse the quality of life.

#### 2.3.6. Observation of Recurrence Rate

Two groups of cured, ineffective, and effective patients were followed up by telephone or outpatient service within 1 month after the end of the course of treatment to investigate whether they had symptomatic recurrence or aggravation, so as to evaluate the recurrence rate of the patients.

### 2.4. Statistical Analysis

All data were processed by SPSS 25.0. The counting data were tested by *χ*^2^ test, the measurement data were expressed by mean ± standard deviation ($\bar{x}\pm \text{s}$), and the *t* test was employed when the variance was uneven. The rank-sum test was adopted for the measurement data and grade data that did not accord with normality. *P* > 0.05 indicates that the difference was not statistically significant, *P* <0.05 indicates that the difference exhibited statistically significant, and *P* < 0.01 was highly statistically significant.

## 3. Results

### 3.1. Comparison of Curative Effect

First of all, we compared the curative effects. The study group was significantly effective in 24 cases, effective in 5 cases, and ineffective in 1 case, and the effective rate was 96.67%. In the control group, 13 cases were markedly effective, 10 cases were effective, and 7 cases were ineffective, and the effective rate was 76.67%. The effective rate of the study group was higher compared to the control group (*P* < 0.05). All the data results are indicated in Figure 1.

RETRACTED

### 3.2. Comparison of Individual Symptom Scores

Secondly, we compared the individual symptom scores. Compared between the two groups, the scores of diarrhea times, stool characteristics, abdominal pain, and abdominal distension in the study group were lower compared to the control group (*P* < 0.05). All the data results are indicated in Table 1.

### 3.3. Comparison of Total Scores of Clinical Symptoms in TCM

Thirdly, we compared the total score of TCM clinical symptoms. Before treatment, there exhibited no significant difference (*P* > 0.05). After treatment, the total score of TCM clinical symptoms decreased. Compared between the two groups, the total score of TCM clinical symptoms in the study group was lower compared to the control group at 1 week, 2 weeks, and 4 weeks after treatment (*P* < 0.05). All the data results are indicated in Table 2.

### 3.4. Comparison of Plasma Gastrointestinal Hormone Levels

Then, we compared the levels of plasma gastrointestinal hormones. Before treatment, there exhibited no significant difference (*P* > 0.05). After treatment, the levels of 5-HT and VIP decreased. The levels of 5-HT and VIP in the study group were lower compared to the control group (*P* < 0.05). All the data results are indicated in Table 3.

### 3.5. IBS-QOL Score Comparison

Then, we compared the scores of IBS-QOL. The scores of anxieties, health worry, behavioral disorder, social reaction, physical intention, interpersonal relationship, dietary concern, and sexual behavior in the study group were significantly lower compared to the control group (*P* < 0.05). All the data results are indicated in Table 4.

### 3.6. Comparison of Recurrence

Finally, we compared the recurrence; the recurrence rate in the study group was lower compared to the control group (*P* < 0.05). All the data results are indicated in Figure 2.

## 4. Discussion

The etiology and pathogenesis of spleen deficiency and dampness exuberant IBS-D are various. If the qi is not transported, the water valley is not assigned, and it is merged with the large intestine, and it will be diarrhea [16]. Yanchun hurt in the wind and cold, from the skin and meridians, into the intestines and stomach, abdominal distension and intestinal ringing, so diarrhea. “Or because of cold, cover cold then gas condensation, unable to operate water valley, so discharge also [16, 17]. “Suwen cited pain” pointed out: “anger is contrary to qi, and even hematemesis and diarrhea.” Xie Xie, the complete book of Jingyue, said, “if you are angry, you will be a cathartic.” It is covered with liver wood and earth, and his temper is injured. Therefore, emotional disorders, annoyance and anger, liver qi discomfort, rebellious spleen, or melancholy thoughts, bad temper, earth deficiency and wood multiplication, or plain spleen deficiency, and eating in anger, but also injuring spleen soil, can cause spleen loss of health, dereliction of duty, clear and turbid, and diarrhea [18]. Among them, dampness is the most important in exogenous evil, and spleen deficiency is the most important in internal injury. It shows that diet and fatigue are easy to damage the spleen and stomach, and the weakness of the spleen and stomach and the internal occurrence of dampness is diarrhea. “Difficult through 57 difficult” cloud: there are five Xiefan, their names are different [19]. Spleen and stomach are the foundation of diarrhea. In the process of disease, external dampness is most likely to hurt the spleen. Spleen deficiency and dampness are easy to cause and affect each other, which makes the transmission of large and small intestine abnormal, imbalance of ascending and descending, clear and turbid. No matter what kind of evil qi is on the basis of injuring the spleen, it can only cause diarrhea when it leads to the loss of healthy movement of the spleen. Therefore, spleen deficiency and dampness are the key factor leading to the occurrence of this disease [20, 21].

RETRACTED

In ancient and modern times, decoction is the most common treatment for IBS-D. Zhang Zhongjing, an ancient physician, who called diarrhea “lower benefit” or “benefit” in his treatise on typhoid and miscellaneous diseases of the treatise on febrile diseases on diarrhea points out: “the reason is in the middle, the middle coke is in the middle, and the benefit lies in the lower coke. Red stone fat Yu surplus grain soup master [22]. The Wuling powder and Zhenwu decoction all reflect the idea of “benefiting urination so real defecation” [23]. The words “diarrhea person” were written by physician Zhu Danxi in Jinkui Hook Xuan. All can move spleen dampness, which makes it clear that diarrhea is mostly caused by exogenous or internal causes of spleen dampness. “Danxi heart method diarrhea”: “wet diarrhea, from sitting in a wet place, so that dampness hurts the spleen, soil cannot control water, there are many of this disease, it is appropriate to remove dampness soup to swallow Wuji pills, supplemented with Weiling decoction.” In the treatment, put forward that more because of dampness, but benefit small water, is the best policy, that is, to urinate, so real defecation [24]. Zhi Ming Zhang Jiebin made it clear that “the treatment of diarrhea is disadvantageous to small water, not its treatment.” Li Dongyuan, a member of the soil-tonifying faction, believes that diarrhea is caused by damage to the spleen and stomach in the final analysis. Li Shicai said wind, wet, hot or cold these four qi can also be catharsis. It is also said that when clearing qi is under, it will give birth to diarrhea, which is also known as the diarrhea of spleen deficiency and depression. Therefore, it is said that most of the dampness becomes five diarrheas [25]. Light osmosis is the most important, so that the dampness goes away from urination. In modern clinic, it is believed that spleen deficiency and dampness is the key to diarrhea. The modern scholar believes that IBS-D is based on spleen deficiency and dampness and is good at using plaster prescription to treat this disease. Take Ganping lukewarm products to tonify the spleen and dissolve dampness without harming the spleen yin. Professor Gan Liming believes that once the spleen is abnormal, its function will inevitably be affected, resulting in the reversion of body water into dampness, grain reverse into stagnation, and clear turbidity mixed with each other, thus leading to diarrhea, so it is mainly caused by spleen deficiency and dampness, which is the root cause of the disease [26]. When the treatment of “dryness and dampness transporting spleen, qi, and stomach” is adopted, Pingwei San can be used to treat it. Professor Fu Zhiquan pointed out that although IBS-D takes spleen deficiency as a disease, it is not limited to spleen deficiency, and its pathogenesis is complex and changeable, often accompanied by clamping or transformation [27]. In addition, dry and wet products such as patchouli, Peran, and Magnolia are often added. Dryness is better than dampness [28]. Modern physicians absorb the treatment ideas of their predecessors and then combine with years of clinical experience to gradually form their own empirical prescription in the treatment. Some scholars gave self-made Xingpi Qushi Yin to treat IBS-D65 cases of spleen deficiency and dampness syndrome [29]. The specific prescription composition is as follows: Codonopsis pilosula, fried Codonopsis, Poria cocos, Astragalus membranaceus, fried Atractylodes macrocephala, alisma alisma, yam, patchouli, Peran, nutmeg, Euryale seed, and roasted licorice. Taking pinaverium bromide tablet alone as the control group, after the course of treatment, it was found that the total effective rate of the treatment group was 92.31%, which was much higher compared to the control group (76.92%), indicating that the clinical effect of self-made Xingpi Qushi Yin in the treatment of spleen deficiency and dampness syndrome IBS-D was satisfactory, and there were no adverse reactions, so it was worth popularizing. According to other scholars' many years of clinical experience, 70 cases of IBS-D patients with spleen deficiency and dampness syndrome were treated with self-made Yichang prescription composed of Radix Paeoniae Alba, Radix Pseudostellariae, fried Coix seed, Fangfeng, Atractylodes macrocephala, Huangzen, tangerine peel, and Coptis chinensis [30]. The treatment can effectively promote the symptoms and signs of digestive tract and enhance the quality of life.

RETRACTED

In the prescription of soothing the liver and invigorating the spleen, Codonopsis pilosula is the king, focusing on invigorating the spleen and replenishing qi, mediating Zhongqi [31]. Auxiliary drugs with Atractylodes macrocephala Koidz and Poria cocos invigorates the spleen and promotes dampness, in order to help the monarch medicine, and improves the curative effect of the monarch medicine, and then, qi and blood are active. “Materia Medica to seek the truth” Yan Fuling “into the four gentlemen, then assisted with the operation to infiltrate the dampness of the spleen home.” The combination of Bupleurum and Radix Paeoniae Alba soothes the liver and relieves depression, collects yin, and helps the monarch medicine to make the spleen and soil healthy, Bupleurum and Radix Paeoniae Alba are compatible with each other and can adjust liver qi, and Bupleurum Shengsan has the disadvantage of “robbing the liver and yin,” while Radix Astragali can tonify Zhongjiao and strengthen the power of tonifying qi. The monarch and minister of the above five medicines share the common tune and the function of liver and spleen [32]. Add Danshen, an important medicine for promoting blood circulation and removing blood stasis, to promote qi, that is, the so-called “qi is the handsome of blood, and blood is the mother of qi”; lentils strengthen the power of diarrhea by invigorating the spleen and relieving diarrhea; Pinellia ternata coincides with tangerine peel, imitating the method of two Chen and stomach regulating qi, so as to eliminate qi stagnation of spleen and stomach, and help Radix Paeoniae Alba and Atractylodes macrocephala to invigorate the spleen and stomach and awaken the spleen and soil [32, 33]. Fructus Aurantii is good at breaking Zhongjiao Qi stagnation, and it is compatible with Atractylodes macrocephala to treat ruffian, Pinellia ternata can eliminate phlegm, tangerine peel is mainly ascending, and Fructus Aurantii and Astragalus membranaceus are to take the opposite method [33]. Licorice can not only reconcile the medicines but also tonify the spleen and replenish qi. Compatibility with tonifying Codonopsis pilosula and Atractylodes macrocephala Koidz is used for spleen deficiency; compatibility with Radix Paeoniae Alba also strengthens the work of relieving pain and relieving pain, acerbity and Yin, and the dryness of various medicines. However, this medicine can help dampness and choke qi, so it should be used with caution for patients with spleen deficiency and internal stagnation of dampness [34]. The main acupoints are Shenque, Tianshu, Daheng, Qihai, Guanyuan, Zhongji, Zhongwan, Xiawan, Shui, and other acupoints [35, 36]. Cross moxibustion connects Ren meridian, Dai pulse, foot Yangming stomach meridian, foot Taiyin spleen meridian, foot Jueyin liver meridian, foot Shaoyin kidney meridian, and other eight and twelve meridians. It expands the scope of indications of the meridians and strengthens the connection between the twelve meridians and the eight odd meridians. Ren pulse is known as the sea of Yin pulse [36]. The Yin essence of the human body, such as essence, blood, and body fluid, plays an important role in regulating the qi and blood of the yin meridian [37]. The belt pulse plays the role of constraining the vertical sutras and strengthens the connection with each other. The moxibustion site stimulates the meridian qi of the stomach meridian of foot Yangming, which is rich in qi and blood. The abdomen is the gathering place of the five internal organs. Zhongwan, Tianshu, Guanyuan, Zhongji, and other acupoints are the acupoints where the qi of the viscera converges in the abdomen. Abdominal moxibustion not only plays the role of proximal treatment of meridians and collaterals but also strengthens the role of meridians by stimulating other meridians [38–40]. Treating IBS-D with the prescription of soothing the liver and invigorating the spleen combined with cross moxibustion, which broadens the single treatment method and gives full play to the advantages of TCM in the treatment of chronic diseases, not only plays a prominent role in relieving clinical symptoms but also plays a positive role in improving the severity of IBS patients [41, 42].

RETRACTED

In summary, the prescription for soothing the liver and invigorating the spleen combined with cross moxibustion has the effect of soothing the liver and invigorating the spleen, resolving dampness and stomach, and can reduce the main clinical symptoms of patients with diarrhea IBS of spleen-stomach damp-heat type, and the overall effect is significant. It can also enhance the emotional state of anxiety and depression and achieve the overall psychological and physical balance and health state, and the recurrence rate is low, so it can be further applied in clinic.

## Figures and Tables

**Figure 1:** Comparison of curative effect between two groups.

**Figure 2:** Comparison of recurrence rate between two groups.

**Table 1:** Comparison of individual symptom scores between the two groups ($\bar{x}\pm s$, points).

Group	*N*	Number of diarrhea	Stool character	Abdominal pain	The stomach is swollen
C group	30	2.31 ± 0.56	2.34 ± 0.55	2.21 ± 0.65	2.45 ± 0.31
R group	30	1.02 ± 0.21	1.04 ± 0.31	1.06 ± 0.22	1.02 ± 0.12
*t*		11.813	11.278	9.178	23.562
*P*		<0.01	<0.01	<0.01	<0.01

**Table 2:** Comparison of the total scores of TCM clinical symptoms between the two groups ($\bar{x}\pm s$, points).

Group	*N*	Before treatment	One week after treatment	2 weeks after treatment	4 weeks after treatment
C group	30	18.59 ± 2.21	15.39 ± 3.31	11.49 ± 1.45	7.29 ± 2.21
R group	30	18.49 ± 2.41	11.92 ± 2.21	8.29 ± 3.31	2.59 ± 1.22
*t*		0.167	4.775	4.850	10.197
*P*		>0.05	<0.01	<0.01	<0.01

**Table 3:** Comparison of 5-HT and VIP levels between the two groups ($\bar{x}\pm s$).

Group	*N*	5-HT		VIP	
		Before treatment	After treatment	Before treatment	After treatment
C group	30	125.85 ± 3.31	104.19 ± 4.31	99.93 ± 2.34	84.92 ± 2.31
R group	30	125.92 ± 3.42	93.96 ± 3.31	99.96 ± 2.46	71.96 ± 3.31
*t*		0.080	10.310	0.048	17.586
*P*		>0.05	<0.01	>0.05	<0.01

**Table 4:** Comparison of IBS-QOL scores between the two groups ($\bar{x}\pm s$, points).

Group	*N*	Anxiety emotion	Behavior disorder	Somatic intention	Social concern	Interpersonal relationship	Health concern	Dietary concern	Sexual behavior
C group	30	2.66 ± 0.31	2.56 ± 0.44	2.56 ± 0.33	2.93 ± 0.32	2.64 ± 0.31	2.16 ± 0.53	2.46 ± 0.21	2.17 ± 0.31
R group	30	1.01 ± 0.11	0.96 ± 0.11	0.93 ± 0.16	1.33 ± 0.31	1.63 ± 0.12	1.24 ± 0.34	1.16 ± 0.31	1.22 ± 0.34
*t*		27.474	19.322	24.343	19.669	16.641	8.002	19.061	11.308
*P*		<0.01	<0.01	<0.01	<0.01	<0.01	<0.01	<0.01	<0.01

## Data Availability

No data were used to support this study.
